# Lignans from *Mosla scabra* Ameliorated Influenza A Virus-Induced Pneumonia via Inhibiting Macrophage Activation

**DOI:** 10.1155/2022/1688826

**Published:** 2022-07-30

**Authors:** Wei Cai, Li-Ren Wu, Shui-Li Zhang

**Affiliations:** ^1^Department of Chinese Materia Medica, Zhejiang Pharmaceutical University, Siming 315100, China; ^2^Zhejiang Laboratory Animal Management Office, Hangzhou Medical College, Hangzhou 310013, China; ^3^Zhejiang Chinese Medical University, Hangzhou 310053, China

## Abstract

The lower respiratory tract infection, induced by influenza virus, coronaviruses, and respiratory syncytial virus, remains a serious threat to human health that can cause a global pandemic. Thus, finding effective chemicals and therapeutic measures to advance the functional restoration of the respiratory tract after infection has been the emphasis of the studies on the subjects. *Mosla scabra* is a natural medicinal plant used for treating various lung and gastrointestinal diseases, including viral infection, cough, chronic obstructive pulmonary disease, acute gastroenteritis, and diarrhoea. In this study, the antiviral and anti-inflammatory effects of total lignans (MSTL) extracted from the plant were investigated in influenza A virus (IAV)-infected mice and RAW 264.7 macrophages. MSTL could not only protect the macrophages against IAV-induced pyroptosis but also could lighten the lung inflammation induced by IAV in vivo and in vitro. The network pharmacology analysis revealed that differentially expressed genes, mainly involving in EGFR tyrosine kinase inhibitor resistance, endocrine resistance, HIF-1 signaling pathway, C-type lectin receptor signaling pathway, and FOXO signaling pathway, contributed to the IAV-induced alveolar macrophage dysfunction. It indicated that MSTL enhanced the function of alveolar macrophages and improved IAV-induced lung injury in mice.

## 1. Introduction

Influenza is an acute respiratory infection caused by influenza viruses, which are highly contagious and have a high incidence. Influenza viruses are classified into three types: A, B, and C. Influenza A virus (IAV) antigens are prone to mutation and have caused many worldwide pandemics, resulting in significant deaths and economic losses worldwide. The high variability of influenza A viruses increases the difficulty of human response to influenza. Since the development and vaccination of preventive vaccines cannot be targeted, the application of anti-influenza drugs has become one of the important means to prevent and treat influenza [1]. Emerging research has demonstrated that in the pathogenesis of influenza virus pneumonia, besides the direct damage caused by a viral infection, immune damage caused by the virus also plays an important role. Among them, alveolar macrophages are the key cells that initiate the inflammatory response in the lung. Influenza virus infection stimulates alveolar macrophages to produce excessive inflammatory factors, inflammatory mediators, and oxygen-free radicals, which intensify the inflammatory response in the lung [2]. Studies show that the lethal consequences of influenza virus infection in mice depend more on immunopathological damage to the host than on direct cellular damage due to virus replication [3–5]. Therefore, blocking macrophage activation is important for the control of influenza virus-induced immune inflammation.

Traditional Chinese medicine (TCM) has a long history of preventing and treating influenza and exerts obvious advantages. [6, 7]. *Mosla scabra*, belonging to the *Lamiaceae* family, is a perennial herb which has been used since the late Han Dynasty for treating and preventing lung and gut diseases, including influenza virus, herpes simplex virus, allergy, and gastroenteritis [8–10]. Previous studies have revealed that *M*. *scabra* flavonoids (MSF), in which the major active compounds were luteolin, apigenin, kaempferol, moslosooflavone I, and moslosooflavone II, inhibited the viral replication in MDCK cells and improved IAV-induced acute lung injury in mice [11–13]. However, after purification by chromatography, the antiviral activities of MSF were lower than its water extract [14, 15], indicating other unknown bioactive compounds in the water extract [16–18]. Several lignans with anti-inflammatory and antiallergic activities had been isolated from the herb and had similar chemical polarities to plant flavonoids [19, 20]. Therefore, we conjectured that those lignans might be other kinds of activity compounds responsible for the therapeutic effects of *M*. *scabra*. In this study, total lignans were prepared from the aerial parts of the plant, and then, their antiviral and anti-inflammatory effects were investigated in IAV-infected MDCK cells and mouse models.

## 2. Materials and Methods

### 2.1. Preparation of Herbal Extracts and Lignan Isolation

The preparation and isolation of the lignans from *M*. *scabra* were employed as previous studies reported [20–22]. About 15 kg of aerial parts of the plant was extracted with 30 L of 95% ethanol 2 times for 24 h by using the heating reflux method. The ethanol extracts were concentrated in the vacuum drier and then separated with petroleum benzene, chloroform, ethyl acetate, and n-butanol in turn. The ethyl acetate extracts loaded on the silica gel were further gradiently eluted by dichloromethane and methanol (1 : 0⟶9 : 1⟶8 : 2⟶7 : 3⟶1 : 1⟶0 : 1) to obtain 4 factions A–D. Both the factions B and C were, respectively, isolated on RP-18 reversed phase column by using 30%, 60%, and 90% methanol. Finally, the elutes derived from 60% methanol of factions B and C were mixed as the total lignans (MSTL).

### 2.2. IAV-Infected Mouse Model and Drug Treatment

Forty-eight male ICR mice (20 g–24 g body weights) were got from Zhejiang Experimental Animal Center. The experiments were approved by the Ethics Committee of Zhejiang Pharmaceutical University. Six groups, namely, control group, model group, positive group (ribavirin, 50 mg/kg), low-dose MSTL-treated (50 mg/kg) group (MSTL50), middle-dose MSTL-treated (100 mg/kg) group (MSTL100), and high-dose MSTL-treated (200 mg/kg) group (MSTL200) were considered in the experiment. Each group had 8 animals. Except for the mice in the control group, other mice were intranasally challenged with a 100-fold dilution of the lung homogenates derived from the IAV-infected mice, which made 90% of infected mice dead [23, 24]. Two hours after infection, those infected mice were orally administrated with different doses of MSTL once a day for 5 days. Five days after viral infection, all the mice were killed after isoflurane anesthesia. The blood of each mouse was obtained for further biochemical analysis. The right lung tissues were soaked into 5 ml of 5% formaldehyde solution, whereas the left lung of each mouse was homogenized for the detection of viral copies by the RT-PCR method as previously reported [25, 26]. The sequences of primers used for the RT-PCR assay are given in Table 1.

The histological characteristics were scored by use the following grading scale: 0 (no), 1 (slight), 2 (moderate), and 3 (severe) [8, 25]. Each part was individually assessed for neutrophil infiltration, alveolar congestion, and interstitial edema. The sum of scores in these 4 parts was explored to present the severity of IAV-induced lung injury.

### 2.3. Detection of Inflammatory Cytokines and Mediators

The blood (200 microliters) of each mouse was added into the tubes and left overnight at 4°C in the refrigerator. Then, serum was obtained, and serum levels of TNF-*α* and IL-1*β* in mice were detected by using the commercialized ELISA kits (Lianke Biotech Co., Ltd., China). Similarly, the levels of proinflammatory cytokines TNF-*α* and IL-1*β* and the inflammation mediators MCP-1, PGE_2_, PLA_2_, and LTB_4_ in cell mediums were detected by ELISA assay.

### 2.4. IAV-Infected Cell Model

The RAW 264.7 cells were inoculated on a 96-well culture plate with a density of 5 × 10^3^ cells/well for 16 h. After the cells adhered to the wall, the original culture medium was discarded and cultured in a serum-free medium for 24 h. Then, the cells were treated with IAV (MOI = 0.8) and lignans alone or in combination for 48 h. After incubation, the cell viability was measured by CCK8 assay [27] to appraise cytotoxicity of MSTL as well as inhibition of IAV replication in vitro.

### 2.5. Flow Cytometry Detection

The cells of each group were washed twice with PBS and then mixed with FITC-labeled caspase-1 staining solution (1 : 30). After incubation for 60 min at 37°C in a 5% CO_2_ incubator, the cells were washed twice with 1 × Wash Buffer and resuspended with PI staining solution (1 : 100). The pyroptotic rates of RAW264.7 cells infected with IAV were detected by flow cytometry (BD, USA).

### 2.6. RT-PCR Detection

Total RNA was extracted from RAW 264.7 cells according to the instructions of the RNA prep pure tissue kit (Tiangen, China). Then, total RNA samples were quantified and stored at −80°C. Specific primers (Table 1) were designed and synthesized by using the TransScript II Green One-Step RT-PCR SuperMix kit in a 20 *μ*l of reaction system under the following conditions: 50°C, 5 min; 94°C, 30 s; 35 cycles of: 94°C, 5 s; 60°C, 30 s. The relative quantification of PCR was performed by using the SybrGreen ER fluorescence detection system (Bio-Rad, USA). The Ct values were normalized by using the housekeeping gene GAPDH as the internal reference. The sequences of primers used for the RT-PCR assay are given in Table 1.

### 2.7. Network Pharmacology Analysis

The network pharmacology analysis was implemented according to the methods represented previously [28–30]. Potential components of MSTL were obtained in the TCMSP database [31] by using drug oral bioavailability (OB) ≥30% and drug-like properties (DL) ≥0.18 as screening conditions. The SMILES strings of the potential components were queried through the PubChem database and entered SwissTargetPrediction web service [32] to obtain protein targets of potential components in MSTL. The keyword “lung inflammation” was entered into the GeneCards database to obtain the target information of lung inflammation-related diseases. The online tool Venny 2.1 was used to intersect the targets of potential components in MSTL with the targets of lung inflammation to obtain the common targets of both. The shared targets were entered into the DAVID database, the species was set as “*Homo sapiens*,” and the rest were kept as default values, for KEGG signaling pathway enrichment analysis was performed. The protein-protein interactions are visualized by using the STRING webservice.

### 2.8. Western Blot Assay

The cells or lung tissues were incubated as abovementioned in Section 2.4. The supernatant in each well was removed, and then, cells were washed with PBS two times and centrifuged at 1000 r/min for 5 min. After discarding the supernatant, the cells were added with 100 *μ*l of RIPA lysate (containing 1 mmol/L PMSF) on ice for 20 min and finally centrifuged at 12000 r/min for 10 min to yield the test samples. About 50 *μ*g of total protein was extracted from each sample, electrophoresed on SDSPAGE, transferred, and closed for 1 h. The antibodies (Proteintech, US) were added and incubated overnight, while secondary antibodies (Proteintech, US) were incubated for 1 h at room temperature. The images were analyzed by Image Lab5.0, and the relative expressions of target proteins were calculated.

### 2.9. Statistical Analysis

The software GraphPad Prism 8.0 was used for data analysis and graphing, and the results were expressed as mean ± SEM. The statistical analysis of multiple groups was performed by using a post hoc test. A value of *P* < 0.05 (two-tailed) was considered statistically significant.

## 3. Results

### 3.1. Total Lignans Protected Mice against IAV-Induced Lung Inflammation

As shown in Figure 1, 5 days after IAV infection, there were obvious pathological changes, such as alveolar congestion, interstitial edema, and neutrophil infiltration, in the lung tissues of the model group, resulting in the biggest pathological scores and highest levels of serum proinflammatory cytokines. Oral administration with MSTL reduced IAV-induced lung inflammation and serum proinflammatory cytokine levels (TNF-*α* and IL-6) in a dose-dependent manner. However, there were no significant differences in viral loads among the model group, low-MSTL-treated group, and middle-MSTL-treated group, indicating the low inhibition of MSTL on the viral replication in vivo.

### 3.2. The Low Inhibition of Lignans from *M*. *scabra* on Viral Replication

As shown in Figure 2, except for ribavirin, treatment with MSTL at the concentration of 2.5–40 *μ*g/ml did not cause significant death of MDCK cells, indicating their low cytotoxicity. Although treatment with 5–40 *μ*g/ml of MSTL significantly increased the cell viabilities of IAV-infected MDCK cells compared with the model group, those protective effects of MSTL were much weaker than ribavirin. Furthermore, inhibitory rates of MSTL on the viral loads of IAV-infected MDCK cells were generally lower than 10%, whereas the rate of ribavirin was about 80%. These results were consistent with the inhibitory effects of MSTL on viral loads in vivo. It indicated that MSTL protected mice against IAV-induced death partly via inhibiting inflammatory response rather than direct viral suppression.

### 3.3. MSTL Reduced the Release of Proinflammatory Mediators in IAV-Infected RAW 264.7 Cells

As shown in Figure 3, treatment with MSTL at the concentrations of 1–15 *μ*g/ml could not cause obvious cell death, but the cell viabilities were dramatically decreased when the treated concentrations were higher than 20 *μ*g/ml. Thus, in this study, 15 *μ*g/ml was considered the biggest nontoxic concentration of MSTL for further analysis. Treatment with 5–15 *μ*g/ml of MSTL could concentration-dependently reduce the pyroptosis of IAV-infected macrophages and the excess secretion of MCP-1, TNF-*α*, IL-1*β*, MCP-1, PGE_2_, PLA_2_, and LTB_4_. Notably, when treated at the same concentration (10 *μ*g/ml), MSTL displayed better inhibition of proinflammatory mediator production than ribavirin, indicating its anti-inflammatory potential.

On the other hand, compared with the control group, IAV infection altered the macrophage phenotype into the M2 subtype, whose surface M2 markers (IL-10 and Arg-1) were highly expressed, while the levels of M1 markers (IL-1*β* and IL-6) were sharply decreased (Figure 4). Intervention with MSTL (5–15 *μ*g/ml) promoted M2-type macrophage polarization through reducing mRNA expressions of M1 phenotype markers (IL-1*β* and IL-6) and increasing M2 markers (IL-10 and Arg-1) in IAV-infected RAW264.7 cells, thereby presenting its obvious anti-inflammatory effects.

### 3.4. Anti-Inflammatory Mechanism of MSTL on IAV-Infected Macrophages

To explore the underlying mechanism of MSTL in IAV-infected RAW 264.7 cells, the target profiles of bioactive compounds in MSTL on IAV-induced lung inflammation were analyzed by network pharmacology. As shown in Figure 5, 132 targets of the main bioactive compounds moslolignan I, moslolignan II, and andamanicin were found to be responsible for the anti-inflammatory effects of MSTL on IAV-infected macrophages. The KEGG analysis showed that all those targets are mainly involved in EGFR tyrosine kinase inhibitor resistance, endocrine resistance, HIF-1 signaling pathway, *C*-type lectin receptor signaling pathway, FOXO signaling pathway, hepatitis B, influenza virus infection, PI3K-Akt signaling pathway, and pathways in cancer. To verify those network pharmacology results, the protein expressions of core genes in host antiviral response and inflammation-related pathways were measured by Western blotting. As expected, IAV significantly increased protein expressions of TLR7, p-p65, p-ERK, p-p38, GSDMD-N, NLRP3, and HIF-1, but decreased protein expressions of p-AKT1 and p-FOXO1 both in the lung tissues of IAV-infected mice and macrophages (Figure 6), which of those trends could be remarkably reversed by MSTL in vivo and in vitro. It demonstrated that MSTL inhibited IAV-induced inflammation in macrophages partly via activation of inflammation-related pathways.

## 4. Discussion

During influenza virus infection, the monocytes/macrophages are recruited from the cycle into the damaged areas of lung tissues to repair the injury and clear the virus, producing and releasing a variety of factors, including proinflammatory cytokines (TNF-*α*, IL-1*β*, and IL-6), antiviral cytokines (IFN-*α*/*γ*) and chemokines (MCP-1), which are directly or indirectly involved in the antiviral response. The immune response induced by these mediators is beneficial to the organism, but if induced excessively, it can be transformed into an immunopathological response, causing destruction of self-cells and inflammatory damage to lung tissues [5, 33–35].

Given the results that MSTL protected mice against IAV-induced death partly via inhibiting inflammatory response rather than direct viral suppression, in this study, we focused on the effects of MSTL on IAV-induced macrophage activation in vitro which was responsible for the initiation of inflammatory cytokine storm. The macrophages have been demonstrated to be involved in all inflammatory diseases. MCP-1 as an important chemokine activates and chemotacticizes alveolar macrophages, playing an important role in the host antiviral response. Likewise, TNF-*α* and IL-1*β* are the important proinflammatory cytokines involved in the host immune and the initiators of the inflammatory response. Numerous animal experiments and clinical trials demonstrated a strong link between their increased circulating levels and host inflammatory response [5, 36]. Viral stimulation can cause activation of PLA_2_, which acts on cell membrane phospholipids to produce arachidonic acid, whose metabolites include leukotrienes (LTs) and prostaglandin products (PGs) [37]. LTB_4_ promotes the antigen-presenting function of dendritic cells, causing local edema through contraction of airway smooth muscle, promotion of mucus secretion, and increase of vascular permeability [38]. PGE_2_ promotes the development of the inflammatory response mainly through its powerful vasodilatation, coactivation of chemokines and attraction of neutrophils, and enhancement of the permeability of the vascular wall [39, 40]. In this study, we found that the levels of MCP-1, TNF-*α*, IL-1*β*, PGE_2_, PLA_2_, and LTB_4_ in the supernatant of alveolar macrophages infected with influenza virus were significantly enhanced, while MSTL significantly inhibited the levels of those proinflammatory cytokines and mediators after virus infection in vitro. Furthermore, MSTL also could reduce the infiltration of inflammatory cells and attenuated the immunopathological damage after IAV infection in mice. However, MSTL hardly inhibits viral replication in vivo and in vitro. These results indicated that MSTL exerted anti-inflammatory potential for prevention of IAV-induced cytokine storm and viral pneumonia, rather than its direct antiviral effects. In addition, the antiviral drug ribavirin was used as the positive control. Although direct inhibitory activities of ribavirin on viral replication could also reduce the production of inflammatory substances after viral infection, the protective mechanism of antiviral drugs did not depend on their anti-inflammatory actions, which were significantly different from MSTL.

Pyroptosis has been demonstrated to be responsible for the fulminant form of macrophage cell death and subsequent release of proinflammatory cytokines [37, 41, 42]. During the process of pyroptosis, GSDMD-N accumulates on the surface of the cell membrane, forming pores of approximately 1.1–2.4 nm in diameter, resulting in a loss of ion concentration balance on both sides of the cell membrane, causing osmotic swelling and lytic death [43]. On the other hand, a large amount of LDH is released from the cells to the extracellular space, and subsequently, many inflammatory substances such as IL-1*β* and IL-18 are also leaked out of the cells. While such a pyroptotic process facilitates the clearance of pathogenic microorganisms and protects against them, the inflammatory response caused by the excessive production of those inflammatory factors is indefinitely amplified, resulting in more serious consequences for the infected organism [44–46]. The results of this study showed that GSDMD-N protein expression was significantly upregulated and caspase-1-mediated cell pyroptosis was significantly increased in IAV-infected macrophages, and MSTL could significantly inhibit IAV-induced macrophage pyroptosis.

The Toll-like receptors (TLRs) are a family of type I transmembrane glycoproteins, which are the major molecules for immune cell recognition of invading pathogens and their products. Among them, TLR3, TLR4, and TLR7 are mainly associated with virus recognition. The ssRNA derived from the influenza virus is recognized by TLR7 and envelope proteins by TLR4, which both activate immune cells by the MyD88-dependent pathway. NF-*κ*B is an important signaling molecule in the TLRs-mediated MyD88-dependent signaling pathway [47–49]. After the activation of the TLR4 or TLR7 signaling pathway, NF-*κ*B inhibitor I*κ*B was degraded and the inhibitory effect on NF-*κ*B was released, and the free NF-*κ*B was translocated into the nucleus and bound to DNA to participate in the transcriptional regulation of various inflammatory factor genes [50]. On the other hand, the viruses hijacked different targeting molecules, such as signaling in FOXO1, HIF-1, and PI3K/AKT pathways, to antagonize nutrition and oxygen deficiency caused by host immune response, thereby replication and immune evasion [51–56]. In this study, network pharmacology and KEGG analysis displayed that the many core molecules in EGFR tyrosine kinase inhibitor resistance, endocrine resistance, HIF-1 signaling pathway, *C*-type lectin receptor signaling pathway, FOXO signaling pathway, hepatitis B, influenza virus infection, PI3K-Akt signaling pathway, and pathways in cancer involved in the anti-inflammatory effects of MSTL in IAV-infected alveolar macrophages. Furthermore, the results of Western blot analysis demonstrated that MSTL downregulated the expressions of TLR7, p-p65, p-ERK, p-p38, GSDMD-N, NLRP3, and HIF-1, but decreased protein expressions of p-AKT1 and p-FOXO1 in both the lung tissues of IAV-infected mice as well as IAV-infected macrophages, indicating the accuracy of bioinformatic results.

In summer, although MSTL could not inhibit IAV-induced viral replication in vivo and in vitro, MSTL could lighten the lung inflammation and proinflammatory mediator production in IAV-infected mice and macrophages. The network pharmacology results revealed that differentially expressed genes, involving in EGFR tyrosine kinase inhibitor resistance, endocrine resistance, HIF-1 signaling pathway, *C*-type lectin receptor signaling pathway, FOXO signaling pathway, hepatitis B, influenza virus infection, PI3K-Akt signaling pathway, and pathways in cancer, contributed to the IAV-induced alveolar macrophage dysfunction. These findings indicated that MSTL enhanced the function of alveolar macrophages and improved outcomes in mice infected with IAV.

## Figures and Tables

**Figure 1:** MSTL ameliorated IAV-induced lung inflammation in mice. (a) The histopathological results of lung tissues observed by the optical microscope (scale bar, 100 *μ*m). (b) The histopathological characteristics scored by using the following grading scale, in which the bigger the score was, the more severity of lung inflammatory response was. (c) The viral loads of the lung tissues detected by qRT-PCR. The average viral loads decreased with increase of Ct values. ND, not detected. (d) The serum levels of TNF-*α* and IL-1*β* detected by ELISA. All data are shown as mean ± SEM (*n* = 8). Different letters meant significant differences (*P* < 0.05) by Tukey's test.

**Figure 2:** Effects of MSTL on viral replication in vitro. (a) Cytotoxicity of MSTL on the proliferation of MDCK cells. (b) Protective effects of MSTL against IAV-induced MDCK cell death. (c) Inhibition of MSTL on the viral loads in IAV-infected MDCK cells. Ribavirin, 10 *μ*g/ml. All data are shown as mean ± SEM (*n* = 5). ND, not detected. Different letters meant significant differences (*P* < 0.05) by Tukey's test.

**Figure 3:** Inhibition of MSTL on IAV-induced pyroptosis and proinflammatory cytokine release of RAW 264.7 cells. (a) Cytotoxicities of MSTL on the proliferation of RAW 264.7 cells. (b) Inhibition of MSTL on IAV-induced pyroptosis of RAW 264.7 cells. (c) Inhibition of MSTL on the release of MCP-1, TNF-*α*, IL-1*β*, PGE_2_, PLA_2_, and LTB_4_ in IAV-infected RAW 264.7 cells. Ribavirin, 10 *μ*g/ml. All data are shown as mean ± SEM (*n* = 5). Different letters meant significant differences (*P* < 0.05) by Tukey's test.

**Figure 4:** MSTL promoted M2-type macrophage polarization by reducing mRNA expressions of M1 phenotype markers (IL-1*β* and IL-6) and increasing M2 markers (IL-10 and Arg-1) in IAV-infected RAW 264.7 cells. The data are presented as the mean ± SEM (*n* = 5). Different letters between the 2 groups indicated the significant difference (*P* < 0.05).

**Figure 5:** The interaction among the targets of bioactive compounds in MSTL. (a) The network of protein-protein interaction. (b) The main pathway contributed to the anti-inflammatory effects of MSTL.

**Figure 6:** Effects of MSTL on the expressions of core proteins in (a) IAV-infected RAW264.7 cells and (b) mice. All data are shown as mean ± SEM (*n* = 5). Different letters meant significant differences (*P* < 0.05) by Tukey's test.

**Table 1:** Sequences of primers used for the RT-PCR assay.

Gene	Primer sequences (5′ to 3′)	Products (bp)
FluA	F: GACCRATCCTGTCACCTCTGAC	235
	R: AGGGCATTYTGGACAAAKCGTCTA	

GAPDH	F: CTCTGGAAAGCTGTGGCGTGATG	120
	R: ATGCCAGTGAGCTTCCCGTTCAG	

IL-1*β*	F: CTA AAGTATGGGCTGGACTG	352
	R: AGCTTCAATGAA AGACCTCA	

IL-6	F: TGATGCACTTGCAGAAAACAA	270
	R: GGTCTTGGTCCTTAGCCACTC	

IL-10	F: TGAATTCCCTGGGTGAGAAGCTGA	147
	R: TGGCCTTGTAGACACCTTGGTCTT	

Arg-1	F: GTGCGATATGCTAGTGGC	180
	R: ATGGTATAGTCCACTGAG	

## Data Availability

The data used to support the findings of this study are included within the article.
